This article has been retracted.

# Histones-Mediated Lymphocyte Apoptosis during Sepsis Is Dependent on p38 Phosphorylation and Mitochondrial Permeability Transition

**DOI:** 10.1371/journal.pone.0077131

**Published:** 2013-10-22

**Authors:** Zhan-Guo Liu, Shu-Yuan Ni, Gui-Ming Chen, Jing Cai, Zhen-Hui Guo, Ping Chang, Yu-Sheng Li

**Affiliations:** 1 Department of ICU, Southern Medical University, Zhujiang Hospital, Guangzhou, China; 2 Department of ICU, The Third Affiliated Hospital of Guangzhou Medical University, Guangzhou, China; 3 Guangdong Provincial Key Laboratory of Geriatric Infection and Organ Function Support, Department of Medical Intensive Care Unit, General Hospital of Guangzhou Military Command, Guangzhou, China; 4 Department of Pathophysiology, Southern Medical University, Guangzhou, China; University of Cincinnati, United States of America

## Abstract

Lymphocyte apoptosis is one reason for immunoparalysis seen in sepsis, although the triggers are unknown. We hypothesized that molecules in plasma, which are up-regulated during sepsis, may be responsible for this. In this study, peripheral lymphocyte apoptosis caused by extracellular histones was confirmed both in mouse and human primary lymphocytes, in which histones induced lymphocyte apoptosis dose-dependently and time-dependently. To identify which intracellular signal pathways were activated, phosphorylation of various mitogen-activated protein kinases (MAPKs) were evaluated during this process, and p38 inhibitor (SB203580) was used to confirm the role of p38 in lymphocyte apoptosis induced by histones. To investigate the mitochondrial injury during these processes, we analyzed Bcl2 degradation and Rhodamine 123 to assess mitochondrial-membrane stability, via cyclosporin A as an inhibitor for mitochondrial permeability transition (MPT). Then, caspase 3 activation was also checked by western-blotting. We found that p38 phosphorylation, mitochondrial injury and caspase 3 activation occurred dose-dependently in histones-mediated lymphocyte apoptosis. We also observed that p38 inhibitor SB203580 decreased lymphocyte apoptotic ratio by 49% (P<0.05), and inhibition of MPT protected lymphocytes from apoptosis. Furthermore, to investigate whether histones are responsible for lymphocyte apoptosis, various concentrations of histone H4 neutralization antibodies were co-cultured with human primary lymphocytes and plasma from cecal ligation and puncture (CLP) mice or sham mice. The results showed that H4 neutralization antibody dose-dependently blocked lymphocyte apoptosis caused by septic plasma *in vitro*. These data demonstrate for the first time that extracellular histones, especially H4, play a vital role in lymphocyte apoptosis during sepsis which is dependent on p38 phosphorylation and mitochondrial permeability transition. Neutralizing H4 can inhibit lymphocyte apoptosis, indicating that it could be a potential target in clinical interventions for sepsis associated immunoparalysis.

## Introduction

Sepsis causes long-term immunosuppression or immunoparalysis, leading to multiple organ failure (MOF) and possibly death [1]. Although sepsis has been recognized as one of the top causes of mortality worldwide, its incidence is continuing to rise dramatically, with approximately 1,400 deaths/day worldwide [2]. Severe sepsis or septic shock is one of the leading causes of admissions to intensive care units. However, there is no specific treatment currently available due to limited understanding of the underlying mechanism behind sepsis [3]. Recently, bundle therapy has been used with barely satisfactory effect, and the costs are high. Hence, further research into the mechanism of sepsis is urgently needed.

It is increasingly being recognized that lymphocyte apoptosis is a vital process in the pathogenesis of sepsis [4], and it is one mechanism of immunosuppression during sepsis, not only because it reduces the number of these critical immune effecter cells [5], but also because of the immunoparalysis caused by apoptotic cells [6]. Moreover, apoptosis of lymphocytes during early stage of sepsis is the major reason for death from this condition [7]. In addition, a reduction in lymphocyte apoptosis is associated with improvement in survival rate in the cecal ligation and puncture (CLP) mouse model [8]. Therefore, understanding the mechanism of lymphocyte apoptosis is crucial for developing effective anti-sepsis therapies [9], [10].

It has been shown that mitogen-activated protein kinases (MAPKs) are involved in the regulation of lymphocyte apoptosis [11], [12]. Furthermore, p38 inhibition is useful for inhibiting lymphoid immunesuppression [13] and improving survival [14] in sepsis. Meanwhile, lymphocyte apoptosis is also mediated by mitochondrial injury [4], [5], [11], [15], resulting in caspase 3 activation [5]. In addition, over-expression of B-cell chronic lymphocytic leukemia/lymphoma 2 (BCL2), which is an anti-apoptosis protein that acts through stabilizing mitochondrial membrane, protects lymphocytes from apoptosis caused by sepsis [16]–[18]. Therefore, the function of components of the MAPK signaling pathway, especially p38, and mitochondrial injury in lymphocyte apoptosis during sepsis are investigated in the present study.

Increases in extracellular histones in the blood of patients with sepsis are associated with prognosis and mortality. Esmon and colleagues reported that levels of extracellular histones were increased in the sera of baboons challenged with *E. coli* and samples collected from patients with sepsis [19], [20]. In addition, histone H4 neutralization antibody has been shown to have a protective effect in various mouse models of sepsis [19], [20]. Furthermore, extracellular histone H4 has been identified as a major antimicrobial component, which induces the death of microbes in the human body [21]. Histones also cause death of endothelial cells during sepsis [20] and induce apoptosis of renal tubular epithelial cells [22].

Based on the above results, we hypothesized that increased levels of extracellular histones are the direct reason for apoptosis of peripheral lymphocytes during sepsis, which results in an irreversible immune dysfunction. These effects may occur through MAPK phosphorylation (especially p38), mitochondrial injury and caspase 3 activation. To confirm this hypothesis, we tested the effect of histones on lymphocytes, and found that histones could lead to lymphocyte apoptosis dose-dependently and time-dependently through p38 phosphorylation, mitochondrial injury and caspase 3 activation. The present study appears to be the first report recognizing a relationship between lymphocyte apoptosis and histone release during sepsis, and addressing the mechanism by which histones induce lymphocyte apoptosis. These results not only add to the understanding of sepsis, but also provide a potential target for anti-immunoparalysis therapies in sepsis.

## Methods

### Reagents

Unless otherwise stated, all the reagents used in this study were purchased from Sigma (St. Louis, MO, USA).

### Animal Model

All animal experiments were approved by the Committee on the Ethics of Animal Experiments of Southern Medical University. Eighteen male mice (8 to 12 weeks old) were randomly separated into three groups (Normal, Sham and CLP). The CLP sepsis mouse model was established following the published protocol [23]. Sham-operated mice underwent operation without ligation and puncture. Un-operated mice were used as the normal group. Plasma or peripheral lymphocytes were harvested 6 h after surgery. Blood of each mouse was too little to separate enough number of lymphocytes for flow-cytometry analysis, so we mixed the lymphocytes of six mice of one group together. Also, we mixed the plasma of the six mice in one group to do the western blotting. And the experiment was repeated three times.

### Human Subjects

Ethical approval was given by the Committee on the Ethics of Experiments of Southern Medical University and all participants provided written informed consent. Peripheral venous blood was taken from three healthy volunteers aged between 20 and 30 years old for each experiment, and was collected into vacuum tubes containing dried lithium heparin. Lymphocytes were separated immediately after collection.

### Separation and Stimulation of Lymphocytes

Lymphocytes were separated from heparinized whole blood using a lymphocyte separation medium (MP Biomedicals, Santa Ana, CA, USA) in accordance with the manufacturer’s instructions. Separated lymphocytes were cultured at a concentration of 1×10^6^/ml in a 96-well plate at 37°C with 5% CO_2_, and were treated with various concentrations (0, 50, 100, 200 µg/ml) of histones (VWR International, Radnor, PA, USA) for a set time (2 h), or were treated with a set concentration (100 µg/ml) of histones for various time durations (0, 2 and 3 h). After incubation, the lymphocytes were collected for analysis of apoptosis, p38 phosphorylation, mitochondrial injury and caspase 3 activation. Inhibitor of p38 activation (25 or 10 µmol/L SB203580) or dimethyl sulfoxide (DMSO) was incubated together with 100 µg/ml histones for 2 h, and then the peripheral lymphocyte apoptotic ratios were tested. Inhibitor of mitochondrial permeability transition, cyclosporin A (CSA) (25 ng/ml or 50 ng/ml), was pre-incubated with human peripheral lymphocytes for 12 h, and then the cells were treated with 50 µg/ml histones for 3 h. Finally, the peripheral lymphocyte apoptotic ratios were tested. To assess extracellular histone H4 neutralization, 20 µl of plasma from CLP mice (which contained histones) or sham mice was co-incubated with various concentrations (0, 10, 25 µg/ml) of H4 neutralization antibody (Cell Signaling Technology, Danvers, MA, USA) for 20 minutes at room temperature. Then plasma from each group was added to the supernatant of isolated human lymphocytes for 2 h, which was followed by flow-cytometry analysis.

### Animal Treatment

Twelve male mice (8 to 12 weeks old) were randomly separated into two groups. The mice were injected with phosphate-buffered saline (PBS) or histones (60 mg/kg weight) through the caudal vein. Whole blood was taken 6 h after injection and lymphocytes were separated for apoptotic ratio analysis.

### Flow-cytometry Analysis

For detection of apoptosis by flow-cytometry analysis, treated lymphocytes were stained with Annexin V and propidium iodide (PI) (BD, Franklin Lakes, NJ, USA) following the manufacturer’s instructions.

### Detection of Mitochondrial Injury

Rhodamine 123 (Rho123) was used for mitochondrial injury detection in accordance with the manufacturer’s handbook.

### Immunoblotting

Using our previously published protocol [24], we used primary antibodies against histone H4, p38, phosphorylated p38 (p-p38), glyceraldehyde 3-phosphate dehydrogenase (GAPDH) and Bcl2 (Cell Signaling Technology, Danvers, MA, USA) followed by incubation with secondary antibodies.

### Statistical Analysis

Data were analyzed using SPSS software (version 13.0; SPSS Inc., Chicago, IL, USA). All data are presented as means ± SD. The differences between experimental and control groups were assessed by the two-tailed unpaired Student’s *t*-test and *p*<0.05 was considered significant.

## Results

### Levels of Extracellular Histone H4 and Peripheral Apoptotic Lymphocytes Increase during the Early Phase of Sepsis in Mice

The sepsis mouse model was established by CLP. Whole blood was collected 6 h later, and the histone H4 level in plasma was tested by western blotting. The result showed that levels of histone H4 in mouse plasma were significantly increased compared with normal or sham group (Fig. 1A). Meanwhile, the peripheral lymphocyte apoptotic ratio (13.11±0.90%) was increased after 6 h in the CLP mice compared with that of normal or sham mice (2.99±0.67%) (Fig. 1B).

**Figure 1:** Lymphocyte apoptotic ratio was increased by extracellular histones in CLP mouse model. A. The levels of plasmic histone H4 of normal, sham or CLP mice were detected by western blotting 6± SD (n = 3). *p<0.05, as compared with normal group. ^‡^ *p*<0.05, as compared with Sham group. C. Histones were injected into mice at the dose of 60 mg/kg weight. Lymphocytes were separated from whole blood 6 h after injection for apoptosis analysis by flow-cytometry. Values are presented as means ± SD (n = 6). *p<0.05, as compared with PBS group.

### Intravenous Injection of Histones Induces Peripheral Lymphocyte Apoptosis in Mice

To test if increased extracellular histone H4 and peripheral apoptotic lymphocytes are interdependent events during sepsis, we injected histones into the caudal vein of anesthetized mice. The peripheral lymphocyte apoptotic ratio was increased by 11.59±0.99% compared with that of the PBS group 6 h after injection (Fig. 1C).

### Histones are Associated with the Apoptosis of Human Peripheral Lymphocytes in Dose-dependent and Time-dependent Manner

The in-vivo mouse experiment showed that extracellular histones, which were increasingly released during sepsis, could induce apoptosis of peripheral lymphocytes. In order to confirm the effect of extracellular histones and expound the mechanisms by which histones induce lymphocyte apoptosis in patients with sepsis, we cultured isolated human lymphocytes with histones *in vitro*. As shown in Fig. 2A, the various concentrations (0, 50, 100, 200 µg/ml) of extracellular histones led to peripheral lymphocyte apoptosis in a dose-dependent manner after 2 h treatment (15.64±2.44%, 77.98±2.90%, 93.61±2.86%, 94.30±3.31%, respectively). Additionally, this dose dependency was mainly correlated with an early apoptotic ratio (7.85±0.53%, 58.14±10.68%, 84.27±6.71%, 85.22±4.72%, respectively). The late apoptotic ratio made no statistically significant difference. Extracellular histones also led to peripheral lymphocyte apoptosis in a time-dependent manner of apoptotic status, but not of a significant ratio. The apoptotic peripheral lymphocytes were largely found to be in early apoptosis (89.54±2.02%) after 2 h of stimulation, but majority found in late apoptosis (91.80±1.54%) after 3 h. The total apoptotic ratios of the two groups were the same (Fig. 2B). Because of this, the early and late apoptotic ratio is not given for other experiments when the composition was the same.

**Figure 2:** Histones induced human lymphocyte apoptosis dose-dependently and time-dependently. Human lymphocytes were cultured with histones of various concentrations (0, 50, 100, 200 µg/ml) or 100 µg/ml histones for various time durations (0, 2, 3 h). Lymphocyes were harvested and apoptotic ratio was detected by flow-cytometry. A. Dose-dependent manner. Values are presented as means ± SD (n = 3). *P<0.05, as compared with 0 µg/ml. ^‡^P<0.05, as compared with 50 µg/ml. B. Time-dependent manner. Values are presented as means ± SD (n = 3). *P<0.05, as compared with 0 µg/ml group.

### Human Peripheral Lymphocyte Apoptosis Associated with Extracellular Histones is p38 Phosphorylation-dependent

To confirm which MAPK signal pathway is necessary for peripheral lymphocyte apoptosis induced by histones, the phosphorylation of p38, ERK and JNK were assessed. The data showed that histones only enhanced the phosphorylation of p38 after 2 h of stimulation (Fig. 3A). The results of ERK and JNK phosphorylation were not shown. The p38 pathways in lymphocytes was blocked by SB203580 after 2 h of incubation. The results showed that SB203580 was able to significantly decrease the peripheral lymphocyte apoptotic ratio (22.21±2.79% vs. 43.83±4.70%) (Fig. 3C).

**Figure 3:** Inhibition of p38 phosphorylation blocked lymphocyte apoptosis induced by histones. A. Western blotting results of P38 phosphorylation. Lymphocytes were harvested after histones treatment for 2± SD (n = 3). ^‡^P<0.05, as compared with 0 µg/ml group. C. Human lymphocytes were exposed to 100 µg/ml histones with DMSO, 10 and 25 µmol/L SB203580. Lymphocyes were harvested 2 h after treatment for apoptosis detection by flow-cytometry. Values are presented as means ± SD (n = 3). *P<0.05, as compared with control.

### Mitochondrial Injury is a Key Mechanism Underlying Histones-mediated Apoptosis in Lymphocytes

Mitochondrial injury plays an important role in the development of lymphocyte apoptosis. Esmon found that histones could cause mitochondrial injury in endothelial cells after injection of histones to mice [20]. Thus, we proposed that mitochondrial injury might be a vital process during histone associated peripheral lymphocyte apoptosis. To confirm this hypothesis, we compared mitochondrial injury in lymphocytes cultured with various concentrations of histones using Rho123 (a dye that reflects the stability of the mitochondrial membrane). Our results showed that histones led to mitochondrial injury dose-dependently (Fig. 4A). And inhibition of mitochondrial permeability transition by CSA could decrease the peripheral lymphocyte apoptosis in a dose dependent manner (Fig. 4D).

**Figure 4:** Mitochondrial injury is a key mechanism to induce histones-mediated apoptosis in lymphocytes. A. Human lymphocytes were cultured with various concentrations (0, 50, 100, 200 µg/ml) of histones. Lymphocyes were harvested 2 h after treatment and mitochondrial injury was detected by flow-cytometry. M5 represent the percentage of lymphocytes without mitochondrial injury. Values are presented as means ± SD (n = 3). *P<0.05, as compared with 0 µg/ml group. B. Western blotting results of Bcl2. Lymphocytes were harvested after histones treatment for 2 h. Equal protein aliquots of cell lysate were examined by immunoblotting with antibodies against GAPDH or Bcl2. GAPDH was used to verify equal gel loading and transblot efficiencies. C. Bar graph of relative Bcl2 intensity. Values are presented as means ± SD (n = 3). ^‡^P<0.05, as compared with 0 µg/ml group. D. Inhibition of mitochondrial permeability transition by CSA (25 and 50 ng/ml) can decrease the peripheral lymphocyte apoptosis. alues are presented as means ± SD (n = 3). ▾ P<0.05, as compared with CSA 0 ng/ml His 50 µg/ml group.

The expression level of Bcl2, a type of anti-apoptosis protein, is another important marker for mitochondrial-membrane stability. We found that the Bcl2 expression level was downregulated after histones stimulation (Fig. 4B).

### Extracellular Histones Activate Caspase 3 during Human Peripheral Lymphocyte Apoptosis

In addition to the mitochondrial pathway, any proapoptotic pathway will eventually trigger caspase 3 activation. Thus, we compared the activation of caspase 3 between three groups treated with various concentrations of histones (0, 50, 100 µg/ml). Using gray-value comparison, we found that histones can cause caspase 3 activation dose-dependently (Fig. 5).

**Figure 5:** Histones induced caspase 3 activation in a dose-dependent manner. A. Isolated human lymphocytes were exposed to various concentrations (0, 50, 100 µg/ml) of histones. Lymphocyes were harvested 1.5 h after treatment and casepase 3 activation was detected by western blotting. Celeaved caspase 3 represents the activation of caspase 3. GAPDH was used to verify equal gel loading and transblot efficiencies. B. Bar graph of relative activated caspase 3 intensity. Values are presented as means ± SD (n = 3). *P<0.05, as compared with 0 µg/ml. ^‡^P<0.05, as compared with 50 µg/ml group.

### Extracellular Histone H4 Neutralization Dose-dependently Reduces Human Peripheral Lymphocyte Apoptosis

We were interested in assessing whether it is possible to inhibit peripheral lymphocyte apoptosis through extracellular histone neutralization, and whether histones are the only reason for lymphocyte apoptosis. In order to standardize our experiments, we co-cultured plasma from CLP mice (containing histones) or sham mice and isolated human lymphocytes with various concentrations of H4 neutralization antibody (0, 10, 25 µg/ml) and control IgG (25 µg/ml). As shown in Fig. 6, the CLP mouse plasma increased the peripheral lymphocyte apoptotic ratio compared with the sham mouse plasma (73.18±2.44% vs. 44.32±5.52%). In addition, the H4 neutralization antibody reduced the peripheral lymphocyte apoptotic ratio in a dose-dependent manner (55.68±2.60% and 35.29±1.34% respectively vs. 73.18±2.44%). Unexpectedly, we found that 25 µg/ml of H4 neutralization antibodies obviously inhibited the peripheral lymphocyte apoptotic ratio caused by the sepsis plasma (35.29±1.34% vs. 44.32±5.52%) (Fig. 6). The histone H4 level in CLP mouse plasma was checked by western blotting (data not shown).

**Figure 6:** Extracellular histone H4 neutralization antibody blocked human peripheral lymphocyte apoptosis induced by plasma of sepsis mouse model dose-dependently. Isolated human lymphocytes were exposed to 20 µl plasma of sham or CLP mice with various concentrations of H4 neutralization antibody (0, 10, 25 µg/ml) and control IgG (25 µg/ml). Lymphocytes were harvested at 2 h and apoptotic ratio was detected by Flow-cytometry. Values are presented as means ± SD (n = 3). *P<0.05, as compared with sham. ^‡^P<0.05, as compared with CLP group. ▾ P<0.05, as compared with CLP+Anti-H4 10 µg/ml group.

## Discussion

Previous data studies have shown that extensive lymphocyte apoptosis occurred in a number of organs [25]–[28], especially in the circulatory system [5], [15], during sepsis. It has also been shown that the peripheral lymphocyte apoptotic ratio increases in the CLP mouse model, which was confirmed by the current study (Fig. 1). However, the triggers of lymphocyte apoptosis during sepsis are yet unknown. Tumor necrosis factor (TNF)-α, which is increased in patients with sepsis [29], can induce apoptosis during sepsis in certain types of cells through a death receptor. However, anti-TNF-α antibodies are unable to block lymphocyte apoptosis in the septic mouse model [30]. Thus, TNF-α couldn’t be the reason for the peripheral lymphocyte apoptosis that occurs during sepsis. In the current study, we first found that extracellular histones were associated with peripheral lymphocyte apoptosis in both mouse (Fig. 1B) and human primary lymphocytes (Fig. 2) in a dose-dependent and time-dependent manner, indicating that extracellular histones are the triggers of this apoptosis. We observed that not only did the extracellular histone H4 neutralization antibody have a dose-dependent effect on inhibition of peripheral lymphocyte apoptosis, but that the appropriate dose could effectively suppress the apoptosis (Fig. 6). These results indicate that extracellular histone H4 is the dominant stimulant for sepsis-related peripheral lymphocyte apoptosis.

Absolute lymphocyte count is decreased not only in sepsis, but also in critically ill patients without sepsis; however, depressed absolute lymphocyte count in sepsis is not the same as that in critically ill patients without sepsis, who can experience a return to normal values quickly. In sepsis, lymphocyte count decreases persistently throughout the course of the disease, which leads to irreversible immunosuppression or immunoparalysis, resulting in serious complications. Identification of extracellular histones inducing peripheral lymphocyte apoptosis presents a model of immunosuppression formation and maintenance, which is like a vicious positive feedback circle (Fig. 7). Histones are released into blood both by the damaged cells in burned, traumatized or surgically operated tissue, and by the dying neutrophils that migrate in increasing numbers into the injured area. Extracellular histones, especially H4, initially induce peripheral lymphocyte apoptosis, as this condition occurs earlier than other types of immunocytes in sepsis [8], [31]. The apoptotic lymphocytes then become the new sources of histones, and these increase the level of extracellular histones in blood. The dramatic rise in extracellular histones activates platelets through toll-like receptor 4 (TLR4) [32], and this may activate neutrophil extracellular traps (NETs) [33], which are another source of histones [19]. In this condition, increased number of neutrophils migrating into the injured area during sepsis is not helpful for patient recovery [8], which has been demonstrated by previous research [34]. In the meantime, professional phagocytes in blood, such as neutrophils, macrophages or certain dendritic cells (DCs), engulf the apoptotic lymphocytes, and this also results in immunosuppression through different pathways [35]–[37]. Consequently, even if the pathogenic factor is removed, extracellular histones can still be released into blood from the apoptotic peripheral lymphocytes and NETs. This results in further failure of lymphocytes, as well as of other immunocytes, such as neutrophils, macrophages or DCs, in which dysfunction occurs either through the phagocytosis of apoptotic cells. Therefore, once infection, burn or trauma occurs to a certain extent, various types of immunocytes are unable to act normally, and the immunosuppressive condition of sepsis maintains itself by a vicious positive feedback circle, unless the extracellular histones and the apoptotic cells are eliminated. This model presents us one of potential mechanisms of immunoparalysis status during sepsis.

**Figure 7:** The immunosuppressive condition of sepsis maintains itself by a vicious positive feedback circle caused by extracellular histones.

The importance of our work lies not only in the identification of extracellular histones as the trigger of peripheral lymphocyte apoptosis, but also indicates possible anti-immunoparalysis targets in sepsis. SB203580, which is a p38 phosphorylation blocker, decreased the peripheral lymphocyte apoptotic ratio from 43.83±4.70% to 22.21±2.79% (Fig. 3C). This indicates that inhibition of p38 phosphorylation is a potential candidate for anti-immunoparalysis therapies through blocking of peripheral lymphocyte apoptosis, as demonstrated by previous research [13], [14]. Inhibition of mitochondrial permeability has a protective function in the septic mouse model [38], and the mechanism may be involved in inhibiting the lymphocyte apoptosis, as shown in the current study. Extracellular histones lead to peripheral lymphocyte apoptosis through mitochondrial injury and inhibition of mitochondrial permeability transition by CSA (Fig. 4). Finally, we found that H4 neutralization antibodies effectively blocked the peripheral lymphocyte apoptosis caused by septic plasma (Fig. 6). This indicates that anti-H4 therapies might be a potential clinical intervention to fight immunoparalysis status of sepsis, which is currently a challenge. Recently, we are carring out in-vivo studies are addressing the effects of anti-H4 therapies on peripheral lymphocyte apoptosis and the functions of other immunocytes during sepsis.
